RETRACTED

# Application of CT Postprocessing Reconstruction Technique in Differential Diagnosis of Benign and Malignant Solitary Pulmonary Nodules and Analysis of Risk Factors

**DOI:** 10.1155/2022/9739047

**Published:** 2022-08-09

**Authors:** Xiaolong Chen, Bingqiang Xu

**Affiliations:** Image Center of Shaanxi Provincial People's Hospital, Xi'an, Shaanxi 710068, China

## Abstract

**Objective:**

To evaluate the application of CT postprocessing reconstruction technique in differential diagnosis of benign and malignant solitary pulmonary nodules and analysis of risk factors.

**Methods:**

A total of 150 solitary pulmonary nodules (SPN) patients admitted to our hospital from January 2020 to January 2022 were selected and divided into the benign SPN group (*n* = 64) and the malignant SPN group (*n* = 86) according to pathological results. All subjects underwent CT plain scan and CT postprocessing reconstruction, and the general information of the subjects was collected. The diagnostic value of CT plain scan and CT postprocessing reconstruction techniques for benign and malignant SPN was compared; and the CT signs of benign and malignant SPN were compared, and the risk factors of malignant SPN were analyzed.

**Results:**

The pathological results of this study showed that there were 64 cases with benign SPN and 86 cases with malignant SPN. The sensitivity, specificity, accuracy, positive predictive rate, and negative predictive rate of CT postprocessing reconstruction technology in diagnosing malignant SPN were 73.44%, 89.53%, 82.67%, 83.39%, and 81.91%, respectively, which were higher than 56.25%, 65.12%, 61.33%, 54.55%, and 66.67% of CT plain scan, and the difference was statistically significant (*P* < 0.05). There were no significant differences in nodule location, nodule density, vacuole sign, vessel convergence, and pleural depression sign between the two groups (*P* > 0.05). There were statistically significant differences in age, nodule diameter, lobulation sign, burr sign, calcification components, and ground-glass components between the two groups (*P* < 0.05). Multivariate analysis showed that age ≥ 60 years, nodule diameter ≥ 15 mm, the presence of lobulation sign, burr sign, ground-glass components, and noncalcification components were independent risk factors for malignant SPN.

**Conclusion:**

CT postprocessing reconstruction technique has high diagnostic value in the differentiation of benign and malignant SPN, age ≥ 60 years, nodule diameter ≥ 15 mm, lobulation signs, burr signs, ground-glass components, and noncalcification components are independent risk factors for malignant SPN.

## 1. Introduction

Solitary pulmonary nodule (SPN) is a class of nodules ≤ 3 cm in diameter that present as a single, well-circumscribed, radiopaque lesion surrounded by air-containing lung tissue, without hilar enlargement, atelectasis, or manifestations of pleural effusion [1]. About 150,000 cases of SPN are detected by screening every year in the world. Among the detected SPNs, malignant tumors account for 10%-70%, 80% of benign lesions are inflammatory granulomas, and 10% are hamartomas [2]. The 5-year survival rate after surgical resection of early-stage lung cancer can be as high as more than 90%, while the 5-year survival rate of middle-advanced lung cancer is less than 5% [3]. The etiology of SPN is not clear, including neoplastic, infectious, inflammatory, vascular or congenital dysplasia diseases, etc. Most of the nodules are benign, and some studies have shown that nearly 50% of SPN will produce malignant lesions. Lung cancer is one of the malignant tumors with the highest clinical morbidity and mortality, so early diagnosis of benign and malignant SPN and treatment will help improve the prognosis of patients [4, 5].

RETRACTED

At present, there are many methods for diagnosing pulmonary nodules: noninvasive examinations such as X-ray, CT, MRI, positron emission computed tomography (PET-CT), fiberoptic bronchoscopy (FOB), and CT-guided percutaneous lung puncture. Invasive examinations include such as video-assisted thoracic surgery (VATS). However, laboratory examinations are mostly negative in the diagnosis of early lung cancer, with insufficient malignant evidence or only as an excluded examination item. Pathological diagnosis is the gold standard for diagnosis of SPN, but pathological diagnosis must obtain lesion tissue, which means invasive [6]. If noninvasive imaging methods can be used to reduce the invasive examination of benign lesions, it is of great clinical significance. The clinical manifestations of SPN are lack of characteristics, and imaging examination is of great significance to judge its benign and malignant lesions. Computed tomography (CT) routine scan, as a noninvasive examination method, has fast imaging speed, high temporal resolution, and spatial resolution and can accurately display the size, location, and shape of lesions. Compared with chest X-ray, CT can detect more nodular lesions, and the axial image of chest X-ray has a single observation surface, which cannot fully reflect the real components of pulmonary nodules [7]. The detection rate of the burr sign, vacuole sign, lobulation sign, air bronchograms, vessel convergence, and pleural depression sign of the patient's lesions by CT routine scan is relatively low [8].

However, CT postprocessing reconstruction technology has fast image processing function and high image quality, can clearly display the anatomical morphology of small lesions, can help doctors observe lesions from multiple angles and understand lesion structure and surrounding tissue structure, and can help improve diagnostic accuracy [9]. In this study, MPR, CPR, MIP, and VR are mainly used in CT postprocessing reconstruction technology. MPR is multiplane reconstruction, which uses cross-sectional volume data to establish two-dimensional tomographic images in coronal, sagittal, and oblique orientations. It can display complex anatomical results of tissues and organs, and the burr and lobulation signs of pulmonary nodules can be clearly displayed on any inclined plane and curved surface, which is significantly better than the traditional axial image and has a good advantage in the display of morphology and invasion scope of lesions [10, 11]. CPR is a special type of MPR, which can observe the relationship between bronchi and pulmonary nodules by using original data after scanning [12]. VR can make full use of the volume data within the scanning volume to obtain real three-dimensional display images with strong spatial three-dimensional sense, which can be used to display the relationship between nodules and their surrounding bronchi, blood vessels, and soft tissues, which can make up for the deficiency of MPR and facilitate the observation of pleural depression sign and vessel convergence [13]. MIP is a technology that uses the highest intense pixels of volume tissue for projection imaging, which reflects the change in density [14]. Therefore, in this study, MPR, CPR, VR, and MIP technologies are combined to obtain clearer images. It can reflect the detailed features of the lesions from multiple angles and directions, which is conducive to the localization and measurement of the lesions and is convenient for doctors to understand the internal density and edge of the lesions and their relationship with small blood vessels, bronchioles, and pleura in the lung, providing reference for the clinical diagnosis of benign and malignant SPN and the formulation of subsequent surgical plans [15, 16]. Based on this, this study used CT postprocessing reconstruction technology to differentiate benign and malignant SPN, explore its diagnostic value, and analyze the risk factors of malignant SPN, in order to provide reference for clinical diagnosis and treatment of SPN.

RETRACTED

## 2. Materials and Methods

### 2.1. Research Subjects

A total of 150 SPN patients admitted to our hospital from January 2020 to January 2022 were selected and divided into benign SPN group (*n* = 64) and malignant SPN group (*n* = 86) according to pathological results. The inclusion criteria are as follows: (1) all patients underwent CT postprocessing reconstruction imaging of pulmonary nodules; (2) SPN was confirmed by pathological results, and it was a single pulmonary nodule; (3) the diameter of nodule is ≤3 cm; (4) the patient's pathological data were complete; and (5) patients who lack of hilar enlargement, atelectasis, or pleural effusion. The exclusion criteria are as follows: (1) patients with history of previous pulmonary surgery, (2) patients with more than one pulmonary nodules in the lung, (3) patients with distant metastasis, (4) patients with previous history of contrast medium allergy, (5) patients with acute infectious diseases, (6) patients with mental disorders or unable to cooperate, (7) patients who dropped out of the study halfway, (8) patients who have received radiotherapy and chemotherapy, and (9) poor CT image quality. This study was approved by the Medical Ethics Committee. In the benign SPN group, there were 14 cases of chronic inflammation, 12 cases of atypical hyperplasia, 8 cases of tuberculosis, 9 cases of hamartoma, 8 cases of inflammatory pseudotumor, 5 cases of lymph node, 4 cases of mechanized pneumonia, 3 cases of bronchiectasis, and 1 case of pneumoconiosis. In the malignant SPN group, there were 77 cases of adenocarcinoma, 3 cases of squamous cell carcinoma, 5 cases of secondary malignant tumor, and 1 case of small cell carcinoma.

### 2.2. Methods

The whole lung scan was performed with Canon Aquilion ONE 640. The patient was placed in supine position, and breath-holding training was performed before the examination. Before the scan, the patient was instructed to take a deep breath and hold his breath. The scanning range was from the entrance of the thorax to the bottom of the lung. Scanning parameters were as follows: tube voltage was 120 kV, tube current was 50 mA, layer thickness was 0.5 mm, layer spacing was 0.5 mm, pitch was 0.984 : 1, and matrix was 256 × 256 mm. Plain scan and enhanced scan using 80 mL iodixanol were performed. In enhanced scanning delay time, threshold triggering technology was adopted, starting from the luminal center at the level of trachea bifurcation of the ascending aorta. When the threshold value of endovascular contrast agent reached 150 HU, the arterial phase scan was automatically triggered with a delay of 6 s, and the venous phase was delayed by 28 s. The original data was input into the workstation. According to the standard reconstruction algorithm, the original chest data obtained after scanning of patients was reconstructed with a thickness of 0.5 mm, and then the obtained image data was transferred to the postprocessing workstation. Three experienced thoracic radiologists performed the following postprocessing on the images: maximum intensity projection (MIP), multiplane reconstruction (MPR), curve planar reconstruction (CPR), and volume rendering (VR). Simultaneously, the principle of blinding was adopted, and the radiologists did not know the grouping of patients. The burr sign, vacuole sign, lobulation sign, air bronchograms, vessel convergence, and pleural depression sign of the patient's lesions were recorded, and the location, shape, and density of nodules were recorded.

RETRACTED

### 2.3. Observation Indicators

General data of patients in both groups were collected, including age, gender, medical history, imaging data, and pathological data. Comparison of the diagnostic value of plain CT scanning and CT postprocessing reconstruction for benign and malignant SPN: the sensitivity, specificity, accuracy, positive predictive value, and negative predictive value of the two methods in diagnosing malignant SPN were analyzed and calculated according to pathological results. Comparison of CT signs between benign and malignant SPN patients: the main imaging signs of benign and malignant SPN were compared, including burr sign, lobulation sign, and vacuole sign, and their independent risk factors were analyzed

### 2.4. Statistical Methods

SPSS 20.0 statistical software was used for statistical analysis; measurement data were expressed as $\bar{x}\pm \text{s}$ and were compared using t test; count data were expressed as rate (%) and were compared using *χ*^2^ test. Multivariate analysis was conducted by binary logistic regression analysis. *P* < 0.05 was considered statistically significant difference.

## 3. Results

### 3.1. Comparison of General Data between the Two Groups

There was a statistically significant difference in age between the two groups (*P* < 0.05); there was no significant difference in other general data between the two groups (*P* > 0.05), as shown in Table 1.

### 3.2. Comparison of CT Signs of Benign and Malignant SPN Patients

There were no significant differences in nodule location, nodule density, vacuolar sign, vessel convergence, and pleural depression sign between the two groups (*P* > 0.05). There were statistically significant differences in nodule diameter, lobulation sign, burr sign, calcification component, and ground-glass component between the two groups (*P* < 0.05), as shown in Table 2.

### 3.3. Independent Risk Factor Analysis of Benign and Malignant SPN Patients

The benign and malignant SPNs (benign = 0, malignant = 1) were taken as dependent variables, and the factors with statistically significant differences among single factors (age, nodule diameter, lobulation sign, burr sign, ground-glass component, and calcification component) were taken as independent variables and assigned values. Age (<60 years = 0, ≥60 years = 1), nodule diameter (<15 mm = 0, ≥15 mm = 1), lobulation sign (no = 0, yes = 1), burr sign (no = 0, yes = 1), ground-glass component (no = 0, yes = 1), and calcification component (yes = 0, no = 1), which were incorporated into the logistic regression model. The regression equation was LogitP = 0.971 × age + 0.749 × nodule diameter + 0.814 × lobulation sign + 1.035 × burr sign + 0.681 × ground‐glass component + 0.834 × calcification component + 0.312. The results showed that age ≥ 60 years, nodule diameter ≥ 15 mm, the presence of lobulation sign, burr sign, ground-glass component, and no calcification component were independent risk factors for malignant SPN. The results are shown in Table 3.

RETRACTED

### 3.4. Comparison of the Diagnostic Value of Plain CT Scan and CT Postprocessing Reconstruction Techniques for Benign and Malignant SPN

The pathological results of this study showed that there were 64 benign SPNs and 86 malignant SPNs. The sensitivity, specificity, accuracy, positive predictive rate, and negative predictive rate of CT postprocessing reconstruction technology in diagnosing malignant SPN were 73.44%, 89.53%, 82.67%, 83.39%, and 81.91%, respectively, which were higher than the 56.25%, 65.12%, 61.33%, 54.55%, and 66.67% of plain CT scan; the differences were statistically significant (*P* < 0.05), as shown in Tables 4 and 5.

### 3.5. CT Images of Patients

As shown in Figure 1, the combination of several techniques can clearly display the lesions in patient with adenocarcinoma (predominantly acinar type).

## 4. Discussion

SPN is a single, opaque, round or round-like lesion with a diameter no larger than 3 cm in the lung and is not accompanied by obstructive pneumonia or atelectasis [17]. Its properties are diverse. Common benign SPNs mainly include inflammatory nodules and tumor-like nodules, while malignant SPNs mainly include lung cancer, carcinoid, tuberculosis, and lymphoma [18, 19]. Benign and malignant diagnosis of SPN is difficult in clinical research. The diagnosis of benign lesions can avoid blind thoracotomy, and the early diagnosis of malignant tumors can effectively improve the survival rate of patients [20]. Early SPN has no obvious symptoms and signs, so its qualitative diagnosis is very important. Chest X-ray is the most convenient and economical method for the diagnosis of SPN, but it has a high rate of missed diagnosis for ground-glass nodules and micronodules [21]. CT is suitable for the screening of lung lesions due to its fast imaging speed and wide scanning range. However, conventional CT scan has a single observation surface and scanning layer thickness is more than 5 mm, which results in poor image display of fine features of pulmonary nodules [22]. With the development of CT technology, its powerful postprocessing reconstruction technology can intuitively display the shape, lobulation, burr, and relationship with blood vessels of intrapulmonary nodules. The stereo sense of CT postprocessing reconstruction technology is strong and can be used as an important supplement of the qualitative diagnosis of SPN, with a wide range of application and simple operation, which makes up for the defect of low spatial resolution of CT tomography images and can effectively improve the diagnosis rate [23].

RETRACTED

The pathological results of this study showed that there were 64 cases with benign SPN and 86 cases with malignant SPN. Univariate analysis showed that there were no significant differences in nodule location, nodule density, vacuolar sign, vessel convergence, and pleural depression sign between the two groups. There were statistically significant differences in age, nodule diameter, lobulation sign, burr sign, calcification component, and ground-glass component between the two groups (*P* < 0.05). Further multivariate analysis found that age ≥ 60 years, nodule diameter ≥ 15 mm, presence of lobulation sign, burr sign, ground-glass component, and no calcification component were independent risk factors for malignant SPN. Age is a common independent risk factor in many benign and malignant prediction models of SPN, and this study is consistent with previous studies [24]. This is mainly due to the decline of patients' physical function and their ability to repair epithelial damage caused by carcinogens as they grow older. Moreover, some patients have underlying diseases, such as chronic bronchitis and tuberculosis, which increase the risk of lung cancer [25]. A retrospective study [26] showed that when the diameter of nodule was <5 mm, 5-10 mm, and >2 cm, the probability of malignancy was <1%, 6%-28%, and 64%-82%, respectively, suggesting that the malignancy rate increased significantly with the increase of nodule diameter. The pathological basis of benign and malignant pulmonary nodules is different, and the occurrence of lobulation sign and burr sign is more likely to be prone to malignant SPN [27]. Lobulation sign is due to the different differentiation degree and growth rate of tumor cells at different parts of tumor edge. It is related to the restriction of lung scaffold structure when tumor grows from inside to outside. On CT, the lesions are presented as arc-shaped protrusions on the surface, which appear to be lobed, and it is more common in adenocarcinoma and squamous cell carcinoma, but less common in benign nodules [28, 29]. Burr sign generally refers to the presence of radial burrs around nodules, short burrs are the most common in malignant nodules, and it has the highest incidence in adenocarcinoma, which is caused by the pulling of surrounding interlobular septa by tumor during growth process, while benign nodules mostly have long burrs [30, 31]. Solid components in ground-glass nodules are mainly caused by the collapse of alveolar cells caused by the invasion and accumulation of tumor cells. The more solid the components in ground-glass nodules, the worse the prognosis [32]. Calcification foci in SPN are mostly benign, suggesting that calcification is mostly caused by healing of old lesions and belongs to stable lesions [33].

RETRACTED

In this study, the sensitivity, specificity, accuracy, positive prediction rate, and negative prediction rate of CT postprocessing reconstruction in diagnosing malignant SPN were 73.44%, 89.53%, 82.67%, 83.39%, and 81.91%, respectively, which were higher than 56.25%, 65.12%, 61.33%, 54.55%, and 66.67% of plain CT scan, suggesting that CT postprocessing reconstruction technique has a high diagnostic value in the differentiation of benign and malignant SPN. Of course, there are some shortcomings in this study. This study is a retrospective study with a small number of patients selected; and the subjects of this study were all patients with high preoperative suspicion of malignant lesions, not all the population, so there was a certain bias in sample selection. Meanwhile, it cannot be compared with MRI and other examination results. In the future, multicenter research will be conducted to expand the sample size to ensure the accuracy of this study.

In conclusion, CT postprocessing reconstruction technology has high diagnostic value in the differential diagnosis of benign and malignant SPN. Age ≥ 60 years, nodule diameter ≥ 15 mm, lobulation sign, burr sign, ground-glass component, and calcification component are independent risk factors for malignant SPN, which can be used as an effective method for early clinical differentiation of benign and malignant SPN.

## Figures and Tables

**Figure 1:** The CT images of a 69-year-old female patient with adenocarcinoma (predominantly acinar type). (a, b) Conventional axial and coronal views (5 mm layer thickness) show subsolid nodules in the apical segment of the right upper lobe (red arrow) with lobulated changes (green arrow). (c, d) Axial reconstruction (1 mm) clearly shows the solid part of the lesion (red arrow) and the ground-glass part (green arrow). (e) Sagittal view of MPR shows the lesion located below the pleura with adjacent pleural thickening (red arrow), and small vacuoles are seen in the lesion (green arrow); (f) shows multiple burrs around the lesion (red arrows), and adjacent pulmonary blood vessels convergence (green arrows); (g) visually shows part of pulmonary blood vessels traversing the lesion (red arrow); (h) stereoscopically shows that the nodule is lobulated (red arrow), with multiple blood vessels in and around the lesion (green arrow).

RETRACTED

**Table 1:** Comparison of general data between the two groups.

Factors	Benign SPN group (*n* = 64)	Malignant SPN group (*n* = 86)	*t*/*χ*^2^	*P*
Gender (cases)				
Male	39 (60.94%)	55 (63.95%)	0.143	0.706
Female	25 (39.06%)	31 (36.05%)		
Age (years)	54.78 ± 10.35	60.11 ± 12.49	2.777	0.006
Smoking history (cases)				
Yes	25 (39.06%)	29 (33.72%)	0.454	0.500
No	39 (60.94%)	57 (66.28%)		
Drinking history (cases)				
Yes	23 (35.94%)	25 (29.07%)	0.795	0.372
No	41 (64.06%)	61 (70.93%)		
Family history of tumor (cases)				
Yes	2 (3.13%)	9 (10.47%)	2.909	0.088
No	62 (96.87%)	77 (89.53%)		
History of COPD (cases)				
Yes	1 (1.56%)	5 (5.81%)	1.727	0.189
No	63 (98.44%)	81 (94.19%)		
History of tuberculosis(cases)				
Yes	1 (1.56%)	7 (8.14%)	3.144	0.076
No	63 (98.44%)	79 (91.86%)		

**Table 2:** Comparison of CT signs of benign and malignant SPN patients.

Factors	Benign SPN group (*n* = 64)	Malignant SPN group (*n* = 86)	*χ* ^2^	*P*
Nodule location				
Left lung	28 (43.75%)	31 (36.05%)	0.913	0.339
Right lung	36 (56.25%)	55 (63.95%)		
Nodule location				
Upper lobe	30 (46.88%)	49 (56.98%)	1.502	0.220
Middle and lower lobes	34 (53.12%)	37 (43.02%)		
Nodule density				
Solid	54 (84.38%)	74 (86.05%)	0.082	0.775
Subsolid	10 (15.63%)	12 (13.95%)		
Nodule diameter (mm)	12.13 ± 0.76	16.04 ± 0.65	33.887	<0.001
Lobulation sign				
Yes	7 (10.94%)	28 (32.56%)	9.588	0.002
None	57 (89.06%)	58 (67.44%)		
Burr sign				
Yes	18 (28.13%)	46 (53.49%)	9.650	0.002
None	46 (71.87%)	40 (46.51%)		
Calcification component				
Yes	20 (31.25%)	2 (2.33%)	24.528	<0.001
None	44 (68.75%)	84 (97.67%)		
Ground-glass component				
Yes	4 (6.25%)	72 (83.72%)	88.105	<0.001
None	60 (93.75%)	14 (16.28%)		
Vacuolar sign				
Yes	0 (0.00%)	7 (8.14%)	3.144	0.076
None	64 (100.00%)	79 (91.86%)		
Vessel convergence				
Yes	3 (4.69%)	10 (11.63%)	2.233	0.135
None	61 (95.31%)	76 (88.37%)		
Pleural depression sign				
Yes	19 (29.69%)	38 (44.19%)	3.274	0.070
None	45 (70.31%)	48 (55.81%)		

**Table 3:** Analysis of independent risk factors in patients with benign and malignant SPNs.

Related factors	*β*	SE	Wald	OR value	95% CI	*P* value
Age	0.971	0.335	8.401	2.641	1.369~5.092	0.004
Nodule diameter	0.749	0.247	9.195	2.115	1.303~3.432	0.003
Lobulation sign	0.814	0.359	5.141	2.257	1.117~4.561	0.024
Burr sign	1.035	0.311	11.075	2.815	1.530~5.179	0.001
Ground-glass component	0.681	0.225	9.161	1.976	1.271~3.071	0.003
Calcification component	0.834	0.121	47.507	2.303	1.816~2.919	<0.001

RETRACTED

**Table 4:** Comparison of the diagnosis results of plain CT scan and CT postprocessing reconstruction techniques for benign and malignant SPN.

	Pathology results		Total
	Benign (*n* = 64)	Malignant (*n* = 86)	
Plain CT scan			
Benign	36	30	66
Malignant	28	56	84
CT postprocessing reconstruction techniques			
Benign	47	9	56
Malignant	17	77	94
Total	64	86	150

**Table 5:** Comparison of the diagnostic efficacy of plain CT scan and CT postprocessing reconstruction techniques for benign and malignant SPN.

	Sensitivity	Specificity	Accuracy	Positive predictive rate	Negative predictive rate
Plain CT scan	56.25% (36/64)	65.12% (56/86)	61.33% (92/150)	54.55% (36/66)	66.67% (56/84)
CT postprocessing reconstruction techniques	73.44% (47/64)^#^	89.53% (77/86)^#^	82.67% (124/150)^#^	83.39% (47/56)^#^	81.91% (77/94)^#^

# indicates *P* < 0.05 when compared with the plain CT scan group.

## Data Availability

The labeled dataset used to support the findings of this study are available from the corresponding author upon request.
